# Dysregulation of circulating miRNAs promotes the pathogenesis of diabetes-induced cardiomyopathy

**DOI:** 10.1371/journal.pone.0250773

**Published:** 2021-04-28

**Authors:** Uzair Ahmed, Usman Ali Ashfaq, Muhammad Qasim, Imtiaz Ahmad, Hafiz Usman Ahmad, Muhammad Tariq, Muhammad Shareef Masoud, Saba Khaliq

**Affiliations:** 1 Department of Bioinformatics and Biotechnology, Government College University, Faisalabad, Pakistan; 2 Department of Physiology and Cell Biology, University of Health Sciences, Lahore, Pakistan; 3 Department of Cardiology, Punjab Institute of Cardiology, Lahore, Pakistan; 4 Department of Biotechnology, Mirpur University of Sciences and Technology, Mirpur, AJK, Pakistan; University of Balochistan, PAKISTAN

## Abstract

Diabetic Cardiomyopathy (DCM) is characterized by myocardial dysfunction caused by diabetes mellitus. After-effects of diabetic cardiomyopathy are far more lethal than non-diabetic cardiomyopathy. More than 300 million people suffer from diabetes and cardiovascular disorder which is expected to be elevated to an alarming figure of 450 million by 2030. Recent studies suggested that miRNA plays important role in the onset of diabetic cardiomyopathy. This study was designed to identify the miRNA that is responsible for the onset of diabetic cardiomyopathy using in silico and in vitro approaches. In this study, to identify the miRNA responsible for the onset of diabetic cardiomyopathy, in silico analysis was done to predict the role of these circulating miRNAs in type 2 diabetic cardiomyopathy. Shared miRNAs that are present in both diseases were selected for further analysis. Total RNA and miRNA were extracted from blood samples taken from type 2 diabetic patients as well as healthy controls to analyze the expression of important genes like AKT, VEGF, IGF, FGF1, ANGPT2 using Real-time PCR. The expression of ANGPT2 was up-regulated and AKT, VEGF, IGF, FGF1 were down-regulated in DCM patients as compared to healthy controls. The miRNA expression of miR-17 was up-regulated and miR-24, miR-150, miR-199a, miR-214, and miR-320a were down-regulated in the DCM patients as compared to healthy controls. This shows that dysregulation of target genes and miRNA may contribute towards the pathogenesis of DCM and more studies should be conducted to elucidate the role of circulating miRNAs to use them as therapeutic and diagnostic options.

## 1. Introduction

Diabetic Cardiomyopathy (DCM) is characterized by heart failure caused by diabetes mellitus without showing any symptoms of ischemia, hypertension, or coronary artery disease [1, 2]. A diabetic Cardiomyopathy is an explicit form of heart failure, which occurs due to the progression of hyperglycemia and hyperinsulinemia independent of other types of heart diseases [3]. The diabetic heart has diastolic dysfunction with preserved ejection fraction that causes pathological remodeling of the heart [4, 5]. More than 300 million people suffer from type 2 diabetes and cardiovascular disorder which is expected to be elevated to the alarming figure of 450 million by 2030 [6, 7]. Type 2 diabetes cases are predicted to rise at the fastest rate in low- and lower-middle-income countries (LMICs). In 2007, over 110 million people in Asia had type 2 diabetes, with a particularly high morbidity and mortality among the young. Asian people with diabetes are at a higher risk of cardio-renal complications due to their young age of onset and long illness duration [8]. The pathogenesis of DCM was not well understood in the past due to its complexity and was discovered recently. Various factors are found to be associated with the onset of DCM including impaired calcium handling, remodeling of extracellular matrix (ECM), increased oxidative stress, altered metabolism, mitochondrial dysfunction, and endothelial dysfunction [6, 9–13]. Some pathways, as well as proteins, were also found to be involved in the onset of DCM like protein kinase C, peroxisome proliferator-activated receptor α (PPAR-alpha), PI3K (phosphatidylinositol 3-kinase), NFκB (nuclear factor-κB), and MAPK (mitogen-activated protein kinase) signaling pathways [14–16].

MicroRNA (miRNA) is a family of short (almost 20–22 nucleotide long), conserved, non-coding, RNAs that regulate the expression of a target gene by binding to 3’UTR (three prime untranslated regions) [17] and resulting in the inhibition of associated signaling pathways [18–20]. Various studies have shown that miRNAs play a crucial role in the regulation of various pathways and can be used as a potential therapeutic agent in the treatment of various diseases like cancer, diabetes, and cardiomyopathies [21]. They can also act as biomarkers to diagnose different diseases but extensive research has to be done to use miRNAs effectively as therapeutic options for the diagnosis and treatment of diseases [22]. Recent studies suggested that miRNA plays an important role in the onset of diabetic cardiomyopathy [12, 13].

The role of miRNA in the onset of cardiomyopathy in type 2 diabetic is poorly understood and very few reports are available. Not a single study is available about the Pakistani population. In this study, we have identified the role of miRNAs in the onset of diabetic cardiomyopathy using _*in silico*_ analysis and confirmed the role of those miRNAs in diabetic cardiomyopathy in the Pakistani patients.

## 2. Materials and methods

### 2.1. miRNA identification

The miRNAs of type 2 diabetes mellitus and cardiomyopathies were identified from HMDD (Human microRNA Disease Database) (http://www.cuilab.cn/hmdd) [23], which is a comprehensive database of miRNA and disease interactions [24]. Then miRNAs, common in the regulation of both diseases were selected. These shared miRNAs are most likely to be involved in the onset of diabetic cardiomyopathy. 50 of miRNAs that were similar in both diseases were identified.

### 2.2. *In silico* target prediction

The literature was reviewed to confirm the targets of these shared miRNA either they affect whole signaling pathways or a certain gene. Moreover, their possible targets were predicted using TargetScanHuman v7.2 (http://www.targetscan.org/vert_72/) [25, 26]. Literature was searched using keywords like miRNA, and diabetic cardiomyopathy using PubMed (https://www.ncbi.nlm.nih.gov/pubmed/). After confirming targets from the literature survey, the targets of miRNAs were predicted through TargetScanHuman v7.2 (http://www.targetscan.org/vert_72/) (Table 1).

**Table 1:** Selected miRNAs based on their targets.

Sr. No	miRNA	Target Genes
**1**	hsa-mir-214	IGF, VEGF, FGF1, ANGP2
**2**	hsa-mir-126	IGF, VEGF, FGF1, ANGP2
**3**	hsa-mir-150	IGF, VEGF, FGF1, ANGP2
**4**	hsa-mir-34a	VEGF, IGF, ANGP2
**5**	hsa-mir-199a	VEGF, IGF, FGF1
**6**	hsa-mir-24	VEGF, IGF, ANGP2
**7**	hsa-mir-320	IGF, VEGF, FGF1, ANGP2
**8**	hsa-mir-17	VEGF, ANGP2

To proceed further and to prove the hypothesis that these miRNAs regulate or play a role in the onset of diabetic cardiomyopathy, wet lab experimentation was designed to evaluate in silico work.

### 2.3. Primer designing

To check the expression level of these genes and miRNAs associated with them, primers were designed for genes as well as miRNAs. For designing primers for genes (IGF, VEGF, FGF1, ANGP2, AKT) Primer3 v4.1.0 (http://bioinfo.ut.ee/primer3/) was used. To design the primers of miRNAs selected above, the sequence of miRNA was downloaded from miRBase (http://www.mirbase.org/) [27]. To design miRNA primers, miRNA Primer Design Tool (http://genomics.dote.hu:8080/mirnadesigntool/index.jsp?action=startpage) [28] was used. All of the designed primers are shown in Table 2.

**Table 2:** Target genes and miRNA primers.

Genes/miRNAs	Forward Primers	Reverse Primers
**VEGF**	TAGAGCTCAACCCAGACACC	ACCAGGCTCCTCTTTGTTCC
**IGF1**	CATGTCCTCCTCGCATCTCT	TGTCTCCACACACGAACTGA
**FGF1**	ACCAATGTGACCTCGACCAT	GCAGCAAACCAGACAGACAA
**ANGPT2**	TGGTTTGATGCATGTGGTCC	GGATCATCATGGTTGTGGCC
**AKT**	ACCTGACCAAGATGACAGCA	CCATCCCTCCAAGCTATCGT
**mir-214**	GTTACAGCAGGCACAGACA	GTGCAGGGTCCGAGGT
**mir-126**	GGGTCGTACCGTGAGTAAT	GTGCAGGGTCCGAGGT
**mir-150**	TTGCTGGTACAGGCCTGG	GTGCAGGGTCCGAGGT
**mir-34a**	GTTTGGCAATCAGCAAGTATAC	GTGCAGGGTCCGAGGT
**mir-199a**	GGGACAGTAGTCTGCACAT	GTGCAGGGTCCGAGGT
**mir-24**	GTTTGGCTCAGTTCAGCAG	GTGCAGGGTCCGAGGT
**mir-320a**	GGGAAAAGCTGGGTTGAGA	GTGCAGGGTCCGAGGT
**mir-17**	GTTACTGCAGTGAAGGCAC	GTGCAGGGTCCGAGGT

### 2.4. Patient enrollment and sampling

The study population consists of 50 type 2 diabetic patients with cardiomyopathy (fasting serum level of peptide C below 0.35 nmol/mL), with long-lasting diabetes mellitus (over 10 years). Age ranged from 30–72 years. A total of 50 apparently healthy control subjects, matched in terms of gender, age, and body mass index (BMI) were also enrolled. A written informed consent was taken from all the participants before the commencement of the study, after ethical approval by the institutional Ethical Review Committee of University of Health sciences, Lahore (UHS/ERC/2020-19). The study protocol is complied with the Helsinki Declaration (7th Revision, October 2013).

The following exclusion criteria were applied: Patients with arterial hypertension, CHD (Coronary heart disease), other diseases, or agents that can affect myocardial function were excluded. Coexisting atrial fibrillation, intra-ventricular blocks, and the cardiac pacemaker was also regarded as the excluding factors.

A blood sample of 3 ml was collected from patients with diabetic cardiomyopathy as well as healthy individuals, through a sterile syringe and added in EDTA containing vacutainer tubes. for total RNA and miRNA extraction, white blood cells (WBCs) and Plasma was isolated using standard protocol. Briefly, to isolate plasma and buffy coat from whole blood firstly, EDTA vacutainers containing blood samples were centrifuged at 4,000 rpm for 10 min at 4°C. This separated plasma from whole blood was collected in a 1.5 ml Eppendorf tube and stored at -20°C. The remaining blood was transferred to 15 ml falcon tubes labeled with sample ID. 10 ml of RBC lysis solution was added into the remaining blood sample and then was centrifuged at 6000 rpm for 15 min at 4°C. The supernatant was discarded and the above step was performed until the pellet containing WBCs or buffy coat became white. This WBC pellet was stored at -20°C for further use.

### 2.5. Total RNA and miRNA isolation

mirVana^TM^ miRNA Isolation Kit (Catalog number: AM1561) by Invitrogen was used to isolate total RNA and miRNA from WBCs and Plasma according to the protocol given by the manufacturer. This kit is capable of extracting both RNA and miRNA from the given sample. The quantity of mRNA and miRNA was checked using Nanodrop 2000 (Catalog number: ND-2000) by Thermo Scientific and the purity of miRNA was assessed by the A_260_/A_280_ value.

### 2.6. cDNA synthesis

RevertAid First Strand cDNA Synthesis Kit (Thermo Scientific) was used to synthesize cDNA of RNA according to the manufacturer’s protocol. The thermal cycler profile for mRNA was set to incubate at 42°C for 60 min and terminate at 70°C for 5 min. cDNA from miRNA was synthesized using miScript II RT Kit (Qiagen) according to the instructions. The thermocycler profile of miRNA was different from the RNA profile and set to incubate at 37°C for 60 min and terminate at 95°C for 5 min. The cDNA of mRNA and miRNA was stored at -20°C. To confirm that our cDNA has been synthesized the cDNA of genes was subjected to polymerase chain reaction by using a housekeeping gene primer like B-Actin or GAPDH followed by 2% agarose gel electrophoresis.

### 2.7. PI3K/AKT Real-time PCR array

To access the regulation and dysregulation of various genes PI3K/AKT pathway was chosen because PI3K/AKT pathway plays important role in the onset of metabolic disorders like diabetes mellitus and DCM. RT^2^ Profiler PCR Array Kit (Catalog number: PAHS-058Z) by Qiagen having PI3K/AKT pathway genes, was used to identify and confirm disease-associated biomarkers and gene expression alterations due to DCM. All samples were pooled for expression array study for PI3k/AKT pathway. The statistical data analysis was done using Qiagen’s RT^2^ Profiler Data Analysis Software. CT values were exported to an Excel file to create a table of CT values. This table was then uploaded on to the data analysis web portal at http://www.qiagen.com/geneglobe. Samples were assigned to controls and test groups. CT values were normalized based on reference genes. This data analysis report was exported from the Qiagen web portal at GeneGlobe.

### 2.8. Gene expression analysis using real-time PCR (QPCR)

Gene-specific primers were used for Real-time PCR analysis of target genes as well as all miRNA genes. The expression levels of target genes and miRNA genes were detected on the CFX96 Real-Time PCR detection system (Catalog number: 1855196) by Bio-Rad using Maxima SYBR Green/ROX qPCR Master Mix (Catalog number: K0222) by Thermo Scientific according to manufacturer’s instructions. Each experiment for relative gene expression was repeated thrice with biological and technical replicates with a set of housekeeping genes B-Actin, GAPDH for selected genes and U6 for miRNA genes. The statistical analysis was done using GraphPad Prism 8.

### 2.9. Correlation between miRNAs and selected genes

The correlation between miRNA and target genes were identified using HMDD (http://www.cuilab.cn/hmdd), TargetScanHuman v7.2 (http://www.targetscan.org/vert_72/) and miRDB (http://www.mirdb.org/). The correlation was depicted using Mindjet Manager 2019 in a network format, which incorporates the expression results from Real-time PCR analysis, literature survey findings, and the results from these online servers.

## 3. Results

### 3.1. Patient demographic data

The study population was consisted of 50 type 2 diabetic cardiomyopathic patients, with long-lasting diabetes mellitus (over 10 years), aged 30–72 years, and 50 non-diseased control subjects, matched in terms of gender, age, and body mass index (BMI). There were 68% men and 34% of women who were subjected to study trials. The mean age of men was 45 and women were 52. Table 3 shows the demographic data of patients.

**Table 3:** Demographic data of patients.

Parameters	Groups	(%)
**Age**	>50 years	49%
	<50 years	51%
**Gender**	Male	68%
	Female	34%
**Diabetes**	Yes	100%
	No	0%
**Myocardial Infarction**	Yes	100%
	No	0%
**Diabetic Family History**	Yes	29%
	No	71%

### 3.2. PIK3/AKT pathway analysis

The cDNA was confirmed by PCR amplification of the housekeeping gene, ACTB, and GAPDH. By using Qiagen RT^2^ Profiler PCR Array Kit, PIK3/AKT pathway was analyzed for the expression of various genes present in the pathway. The expression of various genes was found to be upregulated as well as downregulated during DCM as compared to the control group. Fold-Change (2^ (-Δ ΔCT)) is the normalized gene expression (2^ (-ΔCT)) in the Test Sample divided the normalized gene expression (2^ (-ΔCT)) in the Control Sample. Fold Regulation represents fold-change results in a biologically meaningful way. Fold-change values greater than one indicates a positive- or an up-regulation, and the fold-regulation is equal to the fold-change. Fold-change values less than one indicate a negative or down-regulation, and the fold-regulation is the negative inverse of the fold-change.

The expression of AKT1 and AKT2 was upregulated by 6.74 and 3.30 folds respectively as compared to controls. Whereas, AKT3 and PTEN showed downregulation by -5.37 and -5.20 folds respectively as compared to controls. Table 4 shows the gene in the PIK3/AKT pathway that was found to be upregulated and the number of folds by which they were over-expressed as compared to the control group. Moreover, Table 4 also shows the gene in the PIK3/AKT pathway that was found to be downregulated and the number of folds by which they were over-expressed as compared to the control group.

**Table 4:** Genes in PIK3/AKT pathway which are upregulated and down-regulated in the disease group as compared to the control group.

Up-regulated genes		Down-regulated genes	
Genes	Fold Up-regulation	Genes	Fold Down-regulation
**ADAR**	2.90	**AKT3**	-5.37
**AKT1**	6.74	**EIF2AK2**	-3.33
**AKT2**	3.30	**GSK3B**	-2.56
**CD14**	3.48	**ITGB1**	-3.54
**EIF4B**	2.56	**PIK3CA**	-4.06
**EIF4G1**	6.06	**PIK3CG**	-5.20
**ELK1**	2.30	**PTEN**	-5.20
**FOS**	2.87	**PTK2**	-3.31
**FOXO3**	2.81	**RAC1**	-2.36
**GRB2**	2.44	**RASA1**	-3.98
**HRAS**	11.74	**HPRT1**	-3.69
**HSPB1**	3.75		
**IGF1R**	3.59		
**ILK**	2.71		
**IRAK1**	2.98		
**JUN**	2.42		
**MAPK14**	2.22		
**MAPK3**	2.74		
**MTOR**	4.00		
**NFKBIA**	2.57		
**PDK2**	2.61		
**PDPK1**	2.88		
**PIK3R2**	3.28		
**PRKCA**	2.01		
**PRKCZ**	5.91		
**RAF1**	2.33		
**RHEB**	2.76		
**RPS6KA1**	3.13		
**SHC1**	2.98		
**TOLLIP**	3.00		
**TSC2**	7.07		
**YWHAH**	2.34		

### 3.3. Expression pattern of selected genes

Five target genes including AKT, ANGPT2, FGF1, IGF1, and VEGF were selected for expression analysis. The expression of AKT was found out to be decreased by 0.33 folds in patients than that of its expression in the control group. The expression of ANGPT2 was found out to be increased by 1.77 folds in patients than that of its expression in the control group. The expression of FGF1 was found out to be decreased by 0.48 folds in patients than that of its expression in the control group. The expression of IGF1 was found out to be decreased by 0.13 folds in patients than that of its expression in the control group. The expression of VEGF was found out to be decreased by 0.37 folds in patients than that of its expression in the control group. Whereas, the fold value for the control group was considered as 1. The p-value of all of the selected genes fell in between 0.0001 and 0.0007 by conventional criteria, this difference is considered to be extremely statistically significant. The above data indicate that the expression of ANGPT2 is slightly increased during DCM and expression of AKT, FGF1, IGF1, and VEGF is decreased during the DCM as compared to controls. Fig 1 shows the normalized fold regulation of target genes.

**Fig 1:** Expression pattern of AKT, ANGPT2, FGF1, IGF1, and VEGF during Type 2 diabetic cardiomyopathy. X-axis presenting the target genes along with control and patients’ group. Y-axis is presenting the fold increase or decrease in expression. Error bars indicating the standard deviation from the mean.

### 3.4. Expression pattern of miRNAs

Eight miRNAs including MIR-17, MIR-24, MIR-34a, MIR-126, MIR-150, MIR-199a, MIR-214, and MIR-320a were selected for expression analysis. The expression of MIR-17 was found out to be increased by 1.65 folds in patients than that of its expression in the control group. The expression of MIR-24 was found out to be decreased by 0.33 folds in patients than that of its expression in the control group. The expression of MIR-150 was found out to be decreased by 0.35 folds in patients than that of its expression in the control group. The expression of MIR-199a was found out to be decreased by 0.72 folds in patients than that of its expression in the control group. The expression of MIR-214 was found out to be decreased by 0.37 folds in patients than that of its expression in the control group. The expression of MIR-320a was found out to be decreased by 0.51 folds in patients than that of its expression in the control group. Whereas, the fold value for the control group was considered as 1. MIR-34a and MIR-126 were not detected as in patients having DCM. The p-value of all miRNA genes fell in between 0.0003 and 0.0009 by conventional criteria, this difference is considered to be extremely statistically significant. The above data indicate that the expression of MIR-17 is increased during DCM and expression of MIR-24, MIR-150, MIR-199a, MIR-214, and MIR-320a is decreased during the DCM as compared to controls. Fig 2 shows the normalized fold regulation of miRNAs.

**Fig 2:** Expression pattern of miR-17, miR-24, miR-34a, miR-126, miR-150, miR-199a, miR-214, and miR-320a during type 2 diabetic cardiomyopathy. X-axis presenting the miRNAs along with the control and patients’ group. Y-axis is presenting the fold increase or decrease in expression. Error bars indicating the standard deviation from the mean.

### 3.5. Correlation of miRNAs with selected genes

miR-17 was found out to be up-regulated and correlate with VEGF (down-regulated) and ANGPT2 (up-regulated). miR-24, miR-150, miR-199a, miR-214, and miR-320a were found out to be down-regulated and have a strong correlation with VEGF (down-regulated), AKT (down-regulated), IGF1 (down-regulated), FGF1 (down-regulated), and ANGPT2 (up-regulated). The correlation of miRNAs with target genes are shown in Figs 3 and 4.

**Fig 3:** Correlation of miR-17, miR-24, and miR-150 with the selected genes. The red downward arrow shows the down-regulation of genes and the green upward arrow for the up-regulation of genes.

**Fig 4:** Correlation of miR-199a, miR-214, and miR-320a with selected genes. The red downward arrow shows the down-regulation of genes and the green upward arrow for the up-regulation of genes.

## 4. Discussion

Diabetes mellitus is known to cause micro as well as macrovascular complications in patients which increases the mortality rate significantly [29]. There are various molecular mechanisms involved in the onset of diabetic cardiomyopathy which bears similarity to the mechanisms and alterations identified in failing hearts. Many molecular mechanisms like mitochondrial dysfunction, dysregulation of certain genes, and dysregulation of miRNAs can contribute to the development of diabetic cardiomyopathy [30].

miRNAs (microRNAs) are small non-coding RNAs that are responsible for the post-transcriptional regulation of gene expression. miRNAs can be isolated from tissues as well as bodily fluids like blood and serum and their levels can be detected using qPCR, _*in-situ*_ hybridization arrays, and RNA sequencing [31, 32]. Various studies have shown that miRNAs play a crucial role in the regulation of various pathways and can be used as a potential therapeutic agent in the treatment of various diseases like cancer, diabetes, and cardiomyopathies [21]. They can also act as biomarkers to diagnose different diseases but extensive research has to be done to use miRNAs effectively as therapeutic options for the diagnosis and treatment of diseases [22].

There are many studies present which elucidate the role of tissue-specific miRNAs in animal models, but no study has been done on the role of circulating miRNAs in the prognosis of DCM in humans. The present study focuses on the circulating miRNAs, their isolation, and expression analysis to clarify their possible role in the onset of diabetic cardiomyopathy.

The circulating miRNAs and mRNAs were isolated from blood samples and the specific criteria were followed for sampling. The study population was consisted of 50 type 2 diabetic cardiomyopathic patients, with long-lasting diabetes mellitus (over 10 years), aged 30–72 years, and 50 non-diseased control subjects, matched in terms of gender, age, and body mass index (BMI). There were 68% men and 34% of women who were subjected to study trials. The mean age of men was 45 and women was 52. The p-value of the age was 0.2276 which was considered non-significant. In a similar study, the PIK3/AKT pathway was studied in streptozotocin (STZ) induced diabetic mice and it was found out that AKT was significantly down-regulated during DCM [33].

Expression profiling of target genes AKT, VEGF, IGF1, FGF1, ANGPT2 was done using Real-time PCR in both DCM patients and healthy controls. The expression of ANGPT2 was slightly up-regulated by 1.7 folds in the DCM patients as compared to healthy controls. It shows that abnormal up-regulation of ANGPT2 is somehow associated with the onset of DCM. It has been reported the ANGPT2 expression elevates in STZ induced diabetic mice which in turn causes the pathogenesis of DCM [34–36]. In contrast, the expression level of AKT, VEGF, IGF1, FGF1 were slightly down-regulated by 0.33, 0.37, 0.13, 0.48 folds respectively. It has been reported in various studies that these genes get down-regulated during DCM and by increasing their expression in the heart tissue the effects of DCM can be alleviated significantly [37–48].

Very little information is available on the expression levels of circulating miRNAs in the case of DCM. Expression profiling of miRNAs also showed dysregulation in DCM patients. The expression of miR-17 was found out to be slightly up-regulated by 1.65 folds in patients than that of its expression in the control group. It showed miR-17 overexpresses and can play role in the prognosis of DCM. There is no study present on the circulating miRNAs but a study proved that during DCM the miR-17 is down-regulated in the cardiomyocytes of diabetic mice which is quite different from the results we have obtained in the case of circulating miRNAs [49]. In contrast miR-24, miR-150, miR-199a, miR-214, and miR-320a were slightly down-regulated by 0.33, 0.35, 0.72, 0.37, 0.51 folds, respectively. These results showed that these circulating miRNAs play a crucial role in the development of DCM as compared to healthy controls. Studies suggest miR-24 and miR-214 become down-regulated during DCM and most likely to have a role in the onset of DCM [50, 51], but miR-199a and miR-320a become up-regulated during DCM in heart tissue [52, 53]. Similar to our study, Flower et al., also observed a decreased expression of miR-320 in Asian Indian population with type 2 diabetes, which is frequently present in endothelial cells and controls cell migration and proliferation in response to oxidative stress [54]. Recently, Prado et al. also reported down-regulation of MiR-320a in the plasma of diabetic retinopathy patients compared with Type 2 diabetic patients without retinopathy and healthy subjects [55]. Wang et al. observed decreased expression of miR-199a-3p in patients with T2DM compared with healthy subjects and suggested that reduced miR-199a-3p expression may be associated with protection of vascular endothelial cell injury [56]. In our set of samples, may be both miR-320a and miR-199a serve as regulators of signaling cascade to protect vascular endothelium.

The correlation between miRNA and target genes was identified using HMDD (http://www.cuilab.cn/hmdd), TargetScanHuman v7.2 (http://www.targetscan.org/vert_72/) and miRDB (http://www.mirdb.org/). The results of this study show that upregulation of miR-17 and down-regulation of miR-24, 150, 199a, 214, and 320a dysregulates AKT, VEGF, IGF1, FGF1, and ANGPT2 thus resulting in the onset of DCM. Fig 5 shows the mRNA-miRNA interaction map.

**Fig 5:** mRNA-miRNA interaction map. The upward green arrows show, up-regulation of circulating miRNAs during DCM. The downward red arrows show, down-regulation of circulating miRNAs during DCM. Whereas, the red cross show unavailability of circulating miRNAs during DCM. The red downward arrow shows the down-regulation of genes and the green upward arrow for up-regulation of genes.

These results show that the expression profiling of circulating miRNAs can be different from the tissue-specific miRNAs. There is a dire need to perform more studies on circulating miRNAs to use them as biomarkers for the early diagnosis and to be used as a potential treatment option for DCM.

## Supporting information

S1 Material (DOCX)
